RETRACTED

# Accuracy of Genomic prediction for fleece traits in Inner Mongolia Cashmere goats

**DOI:** 10.1186/s12864-024-10249-7

**Published:** 2024-04-08

**Authors:** Xiaochun Yan, Jinquan Li, Libing He, Oljibilig Chen, Na Wang, Shuai Wang, Xiuyan Wang, Zhiying Wang, Rui Su

**Affiliations:** 1 College of Animal Science, Inner Mongolia Agricultural University, Hohhot, Inner Mongolia Autonomous Region 010018 China; 2 Inner Mongolia Key Laboratory of Sheep & Goat Genetics Breeding and Reproduction, Hohhot, Inner Mongolia Autonomous Region 010018 China; 3 Key Laboratory Of Mutton Sheep & Goat Genetics And Breeding, Ministry of Agriculture And Rural Affairs, Hohhot, Inner Mongolia Autonomous Region 010018 China; 4 Engineering Research Centre for Goat Genetics and Breeding, Inner Mongolia Autonomous Region, Hohhot, Inner Mongolia Autonomous Region 010018 China; 5 Inner Mongolia Jinlai Livestock Technology Co., Ltd, Hohhot, Inner Mongolia Autonomous Region 010018 China; 6 Inner Mongolia Yiwei White Cashmere Goat Co., Ltd, Ordos, Inner Mongolia Autonomous Region 010018 China; 7 Livestock Improvement Center of Alxa Left Banner, Alxa League, Inner Mongolia Autonomous Region 75000 China

**Keywords:** Genomic selection, Fleece traits, Inner Mongolia Cashmere goats, Prediction accuracy, ssGBLUP

## Abstract

The fleece traits are important economic traits of goats. With the reduction of sequencing and genotyping cost and the improvement of related technologies, genomic selection for goats has become possible. The research collect pedigree, phenotype and genotype information of 2299 Inner Mongolia Cashmere goats (IMCGs) individuals. We estimate fixed effects, and compare the estimates of variance components, heritability and genomic predictive ability of fleece traits in IMCGs when using the pedigree based Best Linear Unbiased Prediction (ABLUP), Genomic BLUP (GBLUP) or single-step GBLUP (ssGBLUP). The fleece traits considered are cashmere production (CP), cashmere diameter (CD), cashmere length (CL) and fiber length (FL). It was found that year of production, sex, herd and individual ages had highly significant effects on the four fleece traits (*P* < 0.01). All of these factors should be considered when the genetic parameters of fleece traits in IMCGs are evaluated. The heritabilities of FL, CL, CP and CD with ABLUP, GBLUP and ssGBLUP methods were 0.26 ~ 0.31, 0.05 ~ 0.08, 0.15 ~ 0.20 and 0.22 ~ 0.28, respectively. Therefore, it can be inferred that the genetic progress of CL is relatively slow. The predictive ability of fleece traits in IMCGs with GBLUP (56.18% to 69.06%) and ssGBLUP methods (66.82% to 73.70%) was significantly higher than that of ABLUP (36.73% to 41.25%). For the ssGBLUP method is significantly (29% ~ 33%) higher than that with ABLUP, and which is slightly (4% ~ 14%) higher than that of GBLUP. The ssGBLUP will be as an superiors method for using genomic selection of fleece traits in Inner Mongolia Cashmere goats.

RETRACTED

**Supplementary Information:**

The online version contains supplementary material available at 10.1186/s12864-024-10249-7.

## Introduction

By the end of 2021, the number of goats in stock has been up to 133.32 million in China, and the cashmere yield was about 15,102.18 tons (http://www.stats.gov.cn). Inner Mongolia Cashmere goats (IMCGs) is an important breed of cashmere goats in China, which is famous with its high cashmere yield and excellence quality of cashmere. It is a dual-purpose breed producing cashmere and meat. Reducing cashmere diameter and increasing cashmere yield are the breeding objectives for IMCGs. With the development of quantitative genetics and molecular biology, the selection methods of livestock have been improved gradually[1]. A central methodology is the BLUP method proposed by Henderson in 1975 [2]. Here, genetics parameters can be estimated based on the so-called mixed model equations in which covariance matrices need to be defined. In the standard approach, the pedigree-based relationship matrix (A) is used and the method is referred to as ABLUP. Several studies have demonstrated that using BLUP method can achieve higher genetic gains in pigs compared to individual phenotype selection [3, 4]. Using BLUP method to estimate the breeding value of litter size traits of Landrace pigs, which indicated that selection by BLUP method is feasible for the improvement of the litter size of swine [5]. Jang et al.(2019) assessed that the effect of progeny numbers and pedigree depth on the accuracy of the estimated breeding value (EBV) of Hanwoo beef using BLUP method, the results showed that EBV can show more precise outcome with more progenies [6].

In 2001, the idea of genomic selection (GS) was proposed by Meuwissen. The method can improve estimation accuracy of breeding value, increase genetic gain, in particular by shortening the generation interval and reduce breeding costs[7–10]. Genomic best linear unbiased prediction (GBLUP) utilizes genomic relationships to estimate the genetic merit of an individual [11, 12]. The genomic relationship matrix (**G**) defines the covariance between individuals based on observed similarity at the genomic level, rather than on expected similarity **A** based on pedigree. Thus, more accurate predictions of merit can be obtained. The GBLUP method assigns the same variance to all loci and essentially treats them all as equally important. The single-step genomic BLUP (ssGBLUP) was provided by Legarra et al. [13]. The core idea of ssGBLUP method is to combine pedigree relationship matrix (**A**) and genomic relationship matrix (**G**) to reconstruct a new relationship matrix (**H**) [14–17]. Both, GBLUP as well as ssGBLUP use the same equations as ABLUP, but with different covariance, that is relationship matrices.

RETRACTED

This approach is beneficial for traits that are difficult to measure and traits with low heritability. It has been successfully applied to other livestock, such as dairy cattle [18], beef [19], pigs [20], chickens [21], and sheep [22]. It demonstrated that accuracies of breeding values for milk fatty acid of dairy cattle were low to high, ranging from 0.13 to 0.72 and from 0.18 to 0.74 considering the pedigree and the genomic information, respectively. It was confirmed that the contribution of genomic information in milk yield is more accurate compared to the ABLUP methodology[18]. Zhao (2019) estimated genetic parameters and conducted genomic prediction for five types of sperm morphology abnormalities in a large Duroc boar population by using GBLUP and ssGBLUP method. It showed that the comparative predictive abilities of breeding values with ssGBLUP outperformed that with GBLUP method [20]. Zhu (2021) evaluated the effect of statistical model, heritability and marker density on genomic prediction of six wool traits of sheep. The results showed that the prediction ability of GBLUP model for traits with low heritability was better [22].Muir (2015) reported that the accuracy of GEBV was higher than that estimated by using ABLUP method with simulated data when the enough training generations were provided [23].

Genomic selection has been widely applied in animal breeding programs. However, due to the limitations of sequencing costs, and economic benefits, the application of genome selection for goats has not yet fully developed. With the construction of reference populations and the development of 70 K commercial SNP genotyping chips for goats, a routine application of GS is in sight. In this study, the records of phenotype, genotype, pedigree of 2299 IMCGs was used. Genomic prediction of fleece traits in Inner Mongolia Cashmere goats (IMCGs) using the pedigree based Best Linear Unbiased Prediction (BLUP), Genomic BLUP (GBLUP), single-step GBLUP (ssGBLUP) were performed. This study will provide a reference for genome selection breeding of Inner Mongolia Cashmere goats.

## Materials and Methods

### Phenotypic data

The phenotypic data were collected from an Inner Mongolia YiWei White Cashmere Goat Limited Liability Company, Wulan Town, Etuoke Banner, Ordos City, Inner Mongolia Autonomous Region, China (39°12′N; 107°97′E). In this study, a total of 33,623 production performance records of fleece traits for 2256 individuals (372 males and 1884 females) at ages of 1 to 8 years old were collected from 2011 to 2021. All animal pedigree can be traced back three generations. The fleece traits included cashmere production (CP), cashmere diameter (CD) and cashmere length (CL), fiber length (FL). The basic statistics of phenotypic data were analyzed with Microsoft Excel 2021 (https://www.microsoft.com/zh-cn/microsoft-365/excel) and R4.2.2 (https://www.r-project.org/).

RETRACTED

### Genotype data

The 2299 individuals were genotyped using the Illumina GGP_Goat_70K BeadChip (Illumina, San Diego, CA). Markers on the sex chromosome were discarded. SNPs were selected based on minor allele frequency (MAF > 0.05), proportion of missing genotypes (missing < 0.05), and Hardy Weinberg equilibrium (HWE > 10^–5^). Unqualified SNPs were removed. Moreover, individuals with more than 10% missing genotypes were excluded. Use PLINK1.9 software to perform quality control on genotype data. The genotype data after quality control was utilized to draw the SNP density maps by CMplot packages in R language.

### Estimation of genetic parameters and genomic breeding value

In this study, the fixed effects including sex, year of production, herd (1 to 11), individual age, dam age, birth type were determined by generalized linear model (GLM). The generalized linear model formula was as follow:

1 $$\begin{array}{c}{\mathbf{y}}_{\mathbf{i}\mathbf{j}\mathbf{k}\mathbf{l}\mathbf{m}\mathbf{n}\mathbf{o}}=\mu +{\mathbf{S}}_{\mathbf{i}}+{\mathbf{Y}}_{\mathbf{j}}+{\mathbf{H}}_{\mathbf{k}}+{\mathbf{I}}_{\mathbf{l}}+{\mathbf{D}}_{\mathbf{m}}+{\mathbf{B}}_{\mathbf{n}}+{\mathbf{e}}_{\mathbf{i}\mathbf{j}\mathbf{k}\mathbf{l}\mathbf{m}\mathbf{n}\mathbf{o}}\end{array}$$

where ${{\varvec{y}}}_{{\varvec{i}}{\varvec{j}}{\varvec{k}}{\varvec{l}}{\varvec{m}}{\varvec{n}}{\varvec{o}}}$ is the vector of observations of the animal, ${\varvec{\mu}}$ is the mean value vector of the observations, ${{\varvec{S}}}_{{\varvec{i}}}$ is the effect of sex, ${{\varvec{Y}}}_{{\varvec{j}}}$ is the effect of year of production, ${{\varvec{H}}}_{{\varvec{k}}}$ is the effect of herd, ${{\varvec{I}}}_{{\varvec{l}}}$ is the effect of individual age, ${{\varvec{D}}}_{{\varvec{m}}}$ is the effect of dams of age, ${{\varvec{B}}}_{{\varvec{n}}}$ is the effect of birth type, ${{\varvec{e}}}_{{\varvec{i}}{\varvec{j}}{\varvec{k}}{\varvec{l}}{\varvec{m}}{\varvec{n}}{\varvec{o}}}$ is the effect of residual.

After determining the fixed effect, a repeatability animal model was used to estimate the genetic parameters and genomic breeding values with ABLUP, GBLUP and ssGBLUP methods. All methods were performed by the ASREML software [24].

RETRACTED

In this study, the model was the same for ABLUP, GBLUP and ssGBLUP:

2 $$\begin{array}{c}\mathrm y=\mathbf\mu+\mathbf X\mathrm b+\mathbf Z\mathrm a+\mathbf W\mathrm c+\mathrm e\end{array}$$

where ${\text{y}}$ is the vector of the observations, $\mu$ is the mean value vector of the observations, $b$ is the vector of fixed effects, $a$ is a vector of additive genetic effects, $c$ is a vector of permanent environmental effects and $e$ is a vector of residual. The matrix ${\varvec{X}}$ is the incidence matrix for the fixed effects, ${\varvec{Z}}$ is the incidence matrix relating additive genetic effects and ${\varvec{W}}$ is the incidence matrix relating permanent environmental effects.

In ABLUP, additive genetic effects are sampled from distribution $N(0,{\varvec{A}}{\sigma }_{a}^{2})$; ${{\varvec{\sigma}}}_{{\varvec{a}}}^{2}$ is the additive genetic variance and ${\varvec{A}}$ is the identity by descent (IBD) relationship matrix constructed from pedigree information. In GBLUP, the matrix relating to additive genetic effects for the genomic relationship matrix (**G**) [12, 25]:

3 $$\begin{array}{c}G=\frac{\mathbf{Z}{\mathbf{Z}}^{\mathbf{^{\prime}}}}{2\sum {{\text{p}}}_{{\text{i}}}\left(1-{{\text{p}}}_{{\text{i}}}\right)}\end{array}$$

In ssGBLUP, the matrix relating additive genetic effects for **H** matrix:

4 $$\begin{array}{c}H=\left[\begin{array}{cc}{\mathbf{A}}_{11}-{\mathbf{A}}_{12}{\mathbf{A}}_{22}^{-1}{\mathbf{A}}_{21}+{\mathbf{A}}_{12}{\mathbf{A}}_{22}\mathbf{G}{\mathbf{A}}_{22}^{-1}{\mathbf{A}}_{21}& {\mathbf{A}}_{12}{\mathbf{A}}_{22}^{-1}\mathbf{G}\\ \mathbf{G}{\mathbf{A}}_{22}^{-1}{\mathbf{A}}_{21}& \mathbf{G}\end{array}\right]\end{array}$$

Here,the individuals are divided into two parts: Part 1 contains the individuals whose genotype is not available and Part 2 consists of the phenotype individuals. Thus, ${\mathbf{A}}_{11}$ denotes the entries of $\mathbf{A}$ that provide the relationships within Part 1, ${\mathbf{A}}_{12}$ and ${\mathbf{A}}_{21}$ the relationships between the individuals of the two parts, and ${\mathbf{A}}_{22}$ the pedigree relationships within Part 2. Moreover, ${\mathbf{A}}_{22}^{-1}$ denotes the inverse of${\mathbf{A}}_{22}$.

Construction of the inverse of **H** matrix for ssGBLUP:

5 $$\begin{array}{c}{\mathbf{H}}^{-1}={\mathbf{A}}^{-1}+\left[\begin{array}{cc}0& 0\\ 0& {(\mathbf{G}}^{-1}-{\mathbf{A}}_{22}^{-1})\end{array}\right]\end{array}$$

where ${{\varvec{A}}}^{-1}$ is the inverse matrix of all pedigree relations, ${{\varvec{G}}}^{-1}$ is the inverse matrix of genome relationships, and ${{\varvec{A}}}_{22}^{-1}$ is the inverse matrix of pedigree relations for the genotype individuals.

RETRACTED

### Accuracy of genetic evaluation

In this study, five-fold cross-validation was used to evaluate the accuracy of genomic prediction. Firstly, the individuals were randomly divided into five groups, and then one group was selected as the validation population at each time, and the other four groups were used as the training population. The accuracy of genomic prediction is evaluated by calculating the correlation between the estimated phenotypic value and the true phenotypic value in the validation population divided by the square root of heritability. The formula was as follow:

6 $$\begin{array}{c}{\mathbf{r}}_{{\mathbf{y}}_{\mathbf{i}}{\widehat{\mathbf{y}}}_{\mathbf{i}}}=\frac{\mathbf{c}\mathbf{o}\mathbf{v}\left({\mathbf{y}}_{\mathbf{i}},{\widehat{\mathbf{y}}}_{\mathbf{i}}\right)}{\sqrt{{\mathbf{h}}^{2}}}\end{array}$$

The unbiased of genomic prediction is evaluated by the regression coefficient between the true phenotypic value and the estimated phenotypic value.

7 $$\begin{array}{c}{\mathbf{b}}_{{\mathbf{y}}_{\mathbf{i}}{\widehat{\mathbf{y}}}_{\mathbf{i}}}=\frac{\mathbf{c}\mathbf{o}\mathbf{v}\left({\mathbf{y}}_{\mathbf{i}},{\widehat{\mathbf{y}}}_{\mathbf{i}}\right)}{\mathbf{V}\mathbf{a}\mathbf{r}({\mathbf{y}}_{\mathbf{i}})}\end{array}$$

## Results

### Basic statistical analysis of phenotypic data

Minimums (Min), mean, maximum (Max), standard deviation (SD) and coefficient of variation (CV) values of the fleece traits were presented in Table 1. The averages values of four fleece traits including fiber length, cashmere length, cashmere production, cashmere diameter is 18.89 cm, 6.23 cm, 740.3 g and 15.23 μm, respectively. And the corresponding coefficient of variation were 25.94%, 17.60%, 29.07% and 5.32%. The four fleece traits approximately follow a normal distribution [See Additional file 1, Figure S1].

**Table 1:** The basic statistics of phenotype values of fleece traits in IMCGs

Traits	Mean	Min	Max	SD	CV(%)
FL (cm)	18.89	4.00	35.00	4.90	25.94%
CL (cm)	6.25	1.00	11.00	1.10	17.60%
CP (g)	740.30	100.00	2550.00	215.19	29.07%
CD (μm)	15.23	12.53	18.94	0.81	5.32%

*FL* Fiber Length, *CL* Cashmere Length, *CP* Cashmere Production, *CD* Cashmere Diameter

### Analysis of genotype data

The 43 individuals and 16,360 SNPs were deleted from the raw genotype data. Finally, 2256 individuals and 50,728 markers were used to analyze. The number of SNPs on each chromosome before and after quality control were shown in Fig. 1. The SNP density after quality control were similar over 29 autosomes (Fig. 2).

**Fig. 1:** Comparison of SNP numbers on each chromosome before and after quality control

**Fig. 2:** The distribution of SNP density on each chromosome

RETRACTED

### Determination of fixed effects

The results demonstrated that year of production, sex, herd and individual ages had high significantly effect on the fleece traits (*P* < *0.01*), however, birth type and dams of age had no effect on the fleece traits for FL, CL and CD (*P* > *0.05*) (Table 2). Therefore, year, sex, herd and individual ages should be considered when the genetic parameters of fleece traits in IMCGs were evaluated.

**Table 2:** The fixed effects of fleece traits in IMCGs

Traits	Source	DF	SS	MS	F	*P*-value
FL	Sex	1	4407	4407	214.808	< 0.01
	Year	10	9401	940	45.821	< 0.01
	Herd	12	15,955	1330	64.803	< 0.01
	Individual age	7	3974	568	27.669	< 0.01
	Dams of age	10	370	37	1.804	> 0.05
	Birth type	3	58	19	0.939	> 0.05
	Residuals	9562	196,183	21		
CL	Sex	1	195	194.98	188.052	< 0.01
	Year	10	862	86.2	83.141	< 0.01
	Herd	12	420	34.97	33.723	< 0.01
	Individual age	7	207	29.54	28.494	< 0.01
	Dams of age	10	15	1.45	1.401	> 0.05
	Birth type	3	0	0.05	0.052	> 0.05
	Residuals	9569	9921	1.04		
CP	Sex	1	32,573,794	32,573,794	862.350	< 0.01
	Year	10	18,928,842	1,892,884	50.112	< 0.01
	Herd	12	20,120,019	1,676,668	44.388	< 0.01
	Individual age	7	5,497,610	785,373	20.792	< 0.01
	Dams of age	10	645,407	64,541	1.709	> 0.05
	Birth type	3	701,926	233,975	6.194	< 0.01
	Residuals	8994	339,733,004	37,773		
CD	Sex	1	16.2	16.24	31.918	< 0.01
	Year	4	221.6	55.39	108.859	< 0.01
	Herd	12	506.7	42.22	82.982	< 0.01
	Individual age	7	37.3	5.33	10.474	< 0.01
	Dams of age	10	7.8	0.78	1.538	> 0.05
	Birth type	3	3.3	1.09	2.143	> 0.05
	Residuals	5316	2705.0	0.51		

*P* < 0.01: the difference is extremely significant; *P* < 0.05: the difference is significant; *P* > 0.05: the difference is not significant; *DF *Degree of Freedom, *SS *Sum of Square, *MS *Mean Square

### Estimation of genetic parameters

The residual plots of fleece traits in each method were shown in Figure S2-S4 [See Additional file 1, Figure S2, Figure S3, Figure S4]. All of these indicated that the models fit well. The variance components and genetic parameters of fleece traits in IMCGs were shown in Table 3. The heritability of FL (fiber length), CL (cashmere length), CP (cashmere production) and CD (cashmere diameter) by using ABLUP method were 0.27, 0.06, 0.15 and 0.24 respectively, and the repeatability of FL, CL, CP and CD were 0.51, 0.08, 0.35 and 0.37 respectively. The heritability of FL (fiber length), CL (cashmere length), CP (cashmere production) and CD (cashmere diameter) by using GBLUP method were 0.31, 0.08, 0.20 and 0.28 respectively, and the repeatability of FL, CL, CP and CD were 0.48, 0.08, 0.34 and 0.36 respectively. The heritability of FL, CL, CP and CD by using ssGBLUP method were 0.26, 0.05, 0.15 and 0.22 respectively, and the repeatability of FL, CL, CP and CD were 0.39, 0.05, 0.26 and 0.24 respectively. Because genome information is considered, the heritability estimated by methods GBLUP is higher than that by ABLUP method, and the repeatability estimated is slightly lower. And the standard error of genomic based methods are lower than pedigree.

RETRACTED

**Table 3:** Estimation of genetic parameters of fleece traits in IMCGs

Traits	Method	${\sigma }_{a}^{2}+SE$	${\sigma }_{c}^{2}+SE$	${\sigma }_{e}^{2}+SE$	*h* ^*2*^ + *SE*	*rep* + *SE*
FL	ABLUP	5.68 ± 0.85	4.92 ± 0.63	10.20 ± 0.17	0.27 ± 0.04	0.51 ± 0.01
	GBLUP	6.19 ± 0.60	3.55 ± 0.34	10.22 ± 0.17	0.31 ± 0.02	0.48 ± 0.01
	ssGBLUP	4.28 ± 0.34	2.12 ± 0.37	10.21 ± 0.17	0.26 ± 0.02	0.39 ± 0.01
CL	ABLUP	0.07 ± 0.02	0.02 ± 0.02	0.96 ± 0.02	0.06 ± 0.02	0.08 ± 0.01
	GBLUP	0.09 ± 0.01	0.00 ± 0.00	0.96 ± 0.01	0.08 ± 0.01	0.08 ± 0.01
	ssGBLUP	0.05 ± 0.01	0.00 ± 0.00	0.95 ± 0.01	0.05 ± 0.01	0.05 ± 0.01
CP	ABLUP	6113.01 ± 1178.3	7656.09 ± 997.2	25,697.35 ± 438.6	0.15 ± 0.03	0.35 ± 0.01
	GBLUP	7878.05 ± 912.2	5228.48 ± 635.4	25,885.67 ± 441.9	0.20 ± 0.02	0.34 ± 0.01
	ssGBLUP	5274.59 ± 532.1	3577.87 ± 705.1	25,862.72 ± 441.5	0.15 ± 0.02	0.26 ± 0.01
CD	ABLUP	0.13 ± 0.02	0.07 ± 0.02	0.32 ± 0.01	0.24 ± 0.04	0.37 ± 0.02
	GBLUP	0.14 ± 0.01	0.04 ± 0.01	0.33 ± 0.01	0.28 ± 0.02	0.36 ± 0.02
	ssGBLUP	0.10 ± 0.01	0.01 ± 0.01	0.32 ± 0.01	0.22 ± 0.02	0.24 ± 0.02

${\sigma }_{a}^{2}$ the additive genetic effects variance, ${\sigma }_{c}^{2}$ the permanent environmental effects variance, ${\sigma }_{e}^{2}$ the residual effects variance,  *SE *Standard error, *h* ^2  ^heritability, *rep *repeatability

### Accuracy of GEBV in each method

Akaike's An Information Criterion (AIC) and Schwarz's Bayesian criterion (BIC or SBC) are used to evaluate the effectiveness of model fitting. It was illustrated that the model by using ssGBLUP and GBLUP methods fitted better than that by using ABLUP methods [See Additional file 1, Figure S5]. The accuracy of GEBV by using GBLUP and ssGBLUP methods were shown in Table 4 and Fig. 3. The results demonstrated that the prediction accuracy of four fleece traits by using ssGBLUP and GBLUP were significantly higher than that using ABLUP. The range of predict ability of the fleece traits by using ABLUP, GBLUP and ssGBLUP range are 36.73% ~ 41.25%, 56.18% ~ 69.06%, 66.82% ~ 73.70%, respectively. There was no significant difference in prediction accuracy between the GBLUP and ssGBLUP methods for the other three personality traits, except for CL. Numerically speaking, the prediction accuracy of fleece traits in ssGBLUP method is slightly higher than that in GBLUP method.

RETRACTED

**Table 4:** The accuracy and unbiased of GEBV for fleece traits with three methods

Traits	Method	Accuracy	Accuracyse	Unbiased	Unbiasedse	*P*-value
FL	ABLUP	39.73%^b^	0.0266	1.0096	0.0687	< 0.001
	GBLUP	69.06%^a^	0.0217	1.0643	0.0450	
	ssGBLUP	73.70%^a^	0.0242	1.1006	0.0494	
CL	ABLUP	36.73%^c^	0.0346	1.1865	0.1206	< 0.001
	GBLUP	56.18%^b^	0.0303	1.0724	0.0639	
	ssGBLUP	70.28%^a^	0.0301	1.3182	0.0615	
CP	ABLUP	41.25%^b^	0.0350	1.2106	0.1252	< 0.001
	GBLUP	64.16%^a^	0.0402	1.1740	0.0878	
	ssGBLUP	71.31%^a^	0.0421	1.2190	0.0891	
CD	ABLUP	37.79%^b^	0.0324	0.9592	0.0764	< 0.001
	GBLUP	62.63%^a^	0.0171	1.0853	0.0369	
	ssGBLUP	66.82%^a^	0.0161	1.1040	0.0259	

Note: ^a, b^ represents significant differences. The difference is significant with different letters

**Fig. 3:** Comparison of the accuracy of GEBV for fleece traits with three methods

## Discussion

In this study, the results that sex, year, herd and animal age had highly significant effect on the fleece traits in IMCGs, which is similar to the findings in most studies. Wang (2013) reported that the year of production, sex and herd had highly significant influences on all fleece traits [26]. Salehi (2010) was to evaluate effect of some environmental factors on fiber characteristics of Raeini Cashmere goats, and the results of this study indicated that the fixed effects including age and sex should be considered in the breeding programs[27]. It may be explained by differences in rearing conditions, rainfall, and quality of grassland. In this study, that the results demonstrated that dams of age and birth type had no significant effect on fleece traits of Inner Mongolia Cashmere goats. Newman (1996) found that the dams of age had no significant effect on cashmere diameter and cashmere length on New Zealand cashmere goats [28]. Snyman reported the non-genetic factors affecting the growth and fleece traits of Afrino sheep, in which the dams of age had no significant effect on fiber diameter [29]. Bromley used REML method to estimate the genetic parameters of prolificacy, weight and wool traits of Columbia, Polypay, Rambouillet and Targhee sheep, which illustrated that birth type had no significant effect on fleece traits [30]. However, Zhou reported that the birth type had significant impact on yearling cashmere length, but had no significant impact on cashmere diameter, it is inconsistent with our results [31]. This may be due to the data collection time and the size of the phenotypic data set. Therefore, year, sex, herd and individual ages should be considered when the genetic parameters of fleece traits in IMCGs were evaluated.

RETRACTED

Many methods, including GBLUP, ssGBLUP and Bayesian methods, have been used to perform genomic selection in plants and animals. To some extent, the methods affected the accuracy of the prediction accuracy. The results in this study show that the estimation accuracy of ssGBLUP and GBLUP is significantly higher than that of ABLUP method. It is basically consistent with that in other studies [32, 33]. Mrode (2021) reported that the estimates of heritability for daily milk yield from GBLUP and ssGBLUP were essentially the same [34], which is similar to this study. Lourenco reported that prediction accuracy of GEBV for growth traits and calving ease when using single-step genomic BLUP (ssGBLUP) in Angus cattle was higher than that in using BLUP [35]. Teissier (2019) illustrated that the accuracy of GEBV for milk production traits, udder type traits, and somatic cell scores in French dairy goats was higher than that using other methods. Similarly, the accuracy of GEBV in ssGBLUP for fiber diameter and live body weight was higher than that with other methods in our study [36]. Wei (2020) compared estimates of genetic parameters and the accuracy of breeding values for wool traits in Merino sheep between pedigree-based best linear unbiased prediction and single-step genomic best linear unbiased prediction, the results showed that the heritability of wool traits with ssGBLUP were slightly higher than those obtained with pedigree-based best linear unbiased prediction [37]. The accuracies of estimated breeding values were low to moderate, ranging from 0.362 to 0.573 for the whole population. Compared with ABLUP, GBLUP and ssGBLUP has relatively better prediction ability. Therefore, it is suggested to use ssGBLUP method for genome selection of goats. With the continuous progress of breeding work, more efficient and simple models will be optimized and developed. Applying these methods to perform genomic selection of important traits in livestock and poultry will inevitably accelerate the breeding process of population.

## Conclusions

In this study, the genetic parameters and genomic breeding values of fleece traits in IMCGs were estimated by using ABLUP, GBLUP and ssGBLUP methods. Regardless of which method is used, the heritability of cashmere length is low, while the heritability of other three fleece traits are medium or low to medium. The prediction accuracy of GEBV for fleece traits by using GBLUP and ssGBLUP is significantly higher than that with ABLUP method. And the prediction accuracy of fleece traits in ssGBLUP method is slightly higher than that in GBLUP method. The accuracy of GEBV with ssGBLUP method for fleece traits ranged from 66.82% to 73.70%, which is 29.03%-33.97% higher than that with ABLUP method. Therefore, ssGBLUP is recommended as the method of genetic evaluation of fleece traits in IMCGs.

RETRACTED

### Supplementary Information

**Supplementary Material 1.**

## Data Availability

The original contributions presented in the study are publicly available. Please refer to https://db.cngb.org/, or email: CNGBdb@cngb.org for detailed application guidance. The accession code CNP0005155 should be included in the application.

## Declarations

**Ethics approval and consent to participate.**

The phenotypic data of cashmere goats used in this manuscript were all recorded by Inner Mongolia YiWei White Cashmere Goat Limited Liability Company. The genotype data comes from the previous accumulation of the research group. This study does not involve animal experiments. Not applicable.
